RETRACTED

# Lemierre’s Syndrome: A Case of Life-Threatening Infection From Family Medicine Practice

**DOI:** 10.7759/cureus.20684

**Published:** 2021-12-25

**Authors:** Sultan O Gohal, Ishtiyaq M Alsubhi, Essa A Alharbi, Hashim E Alkhalaf, Bandar H Alnefaie, Raghad A Althomali, Bayan A Hasan, Mada A Alsadi, Assaf H Alamri, Abdulrahman A Alharbi, Meshal Y Almanea, Ftoon S Almarshood, Saleh A Almoallem, Afaf F Albogami, Faisal Al-Hawaj

**Affiliations:** 1 College of Medicine, Batterjee Medical College, Jeddah, SAU; 2 Department of General Practice, King Salman Specialist Hospital, Hail, SAU; 3 College of Medicine, Northern Border University, Arar, SAU; 4 College of Medicine, King Faisal University, Hofuf, SAU; 5 College of Medicine, King Saud bin Abdulaziz University for Health Sciences, Riyadh, SAU; 6 College of Medicine, Arabian Gulf University, Manama, BHR; 7 College of Medicine, Jordan University of Science and Technology, Irbid, JOR; 8 Department of Otolaryngology, King Abdulaziz Hospital, Makkah, SAU; 9 College of Dentistry, Riyadh Elm University, Riyadh, SAU; 10 College of Medicine, Alfaisal University, Riyadh, SAU; 11 College of Medicine, Jouf University, Al-Jawf, SAU; 12 College of Medicine, Taif University, Taif, SAU; 13 College of Medicine, Imam Abdulrahman Bin Faisal University, Dammam, SAU

**Keywords:** case report, lemierre’s syndrome, internal jugular vein thrombophlebitis, acute pharyngitis, antibiotic prescription

## Abstract

The use of antibiotic therapy has led to a major transformation in medicine with a substantial reduction in mortality. Due to the adverse effects associated with inappropriate antibiotic use, antibiotic stewardship interventions have been promoted to improve antibiotic prescription. However, delayed antibiotic therapy, when clinically needed, may result in increased morbidity. Here, we report the case of a previously healthy young man with an untreated acute upper respiratory infection for two weeks, who presented with headache and fever. Physical examination suggested meningitis as evident by neck stiffness and positive Kernig sign. Purulent tonsilitis was also noted. Laboratory findings showed leukocytosis and elevated inflammatory markers. The patient underwent a computed tomography scan to rule out space-occupying lesions prior to lumbar puncture. The scan revealed thrombophlebitis of the left internal jugular vein that extended to the dural venous sinuses. Magnetic resonance imaging confirmed the intracranial dissemination of the disease. Such findings conferred the diagnosis of Lemierre’s syndrome. The patient was admitted to the intensive care unit where he received systemic anticoagulation and prolonged intravenous antibiotics. He developed a good response and was discharged with no residual deficits after six weeks of hospitalization. Lemierre’s syndrome is a serious infection that develops after a pharyngeal infection. Considering the high mortality rate of untreated Lemierre’s syndrome, physicians should keep a high index of suspicion for this condition when they encounter a patient with upper respiratory tract infection with clinical or radiological findings consistent with internal jugular thrombophlebitis.

RETRACTED

## Introduction

The use of antimicrobial drugs had led to a significant transformation in clinical medicine with a major decrease in morbidity and mortality. In the outpatient department, acute respiratory tract infections are the most frequent indication of antibiotic prescriptions [1]. However, the inappropriate use of antibiotic therapy is associated with the risk of side effects, antibiotic resistance, and increased healthcare costs [2]. Antibiotic stewardship includes interventions that promote the optimal use of antibiotics in terms of their choice, dose, and duration of administration [2]. This made the practice of antibiotic prescription more conservative. A recent population-based study found that delayed antibiotic therapy in the outpatient department for acute upper respiratory tract infection was associated with higher rates of hospital admissions [3]. Here, we present a case of a young man with acute upper respiratory tract infection for two weeks who did not receive any antibiotic prescription and developed septic thrombophlebitis involving the internal jugular vein, Lemierre’s syndrome, which is a rare clinical syndrome in the antibiotic era [4].

## Case presentation

A 22-year-old man was brought to our family medicine clinic with a complaint of severe headache and fever. The headache was bilateral and started two days before the presentation. It was stabbing in nature. He described the severity of the pain as nine out of 10 on the severity scale. He was not able to sleep because of the pain. The pain was radiating to the neck and resulting in neck stiffness. He used over-the-counter analgesic medications, but it did not result in a significant improvement. The headache was worsened by being supine. It was associated with nausea and vomiting. No history of weakness, numbness, or loss of consciousness. Two weeks before this headache, the patient had an upper respiratory tract infection. He visited multiple outpatient clinics and he was offered symptomatic treatment only. Such treatment resulted in partial improvement of his symptoms. He was not given antibiotic therapy for his infection. The patient was not known to have any previous comorbid conditions. He had no previous surgical interventions. Apart from multivitamin supplements, he did not use any medications. He had no drug allergies. He never smoked or consumed alcohol. He was single and a college student. The family history was remarkable for inflammatory bowel disease.

RETRACTED

Upon examination, the patient was drowsy. His vital signs showed tachycardia (122 bpm) and fever (38.5℃). The patient had neck stiffness and a positive Kernig sign. However, the neurological examination showed no focal deficits. Examination of the neck showed multiple enlarged cervical lymph nodes. Throat examination showed congested tonsils with pus. Cardiorespiratory examination yielded normal results. Basic laboratory investigations revealed leukocytosis (14,000/μL), elevated C-reactive protein (20.4 mg/dL), and a high level of erythrocyte sedimentation rate (49 mm/hr). Other laboratory findings are summarized in Table 1. These findings are suggestive of an active inflammatory process.

**Table 1:** Summary of the results of laboratory findings

Laboratory Investigation	Result
Hemoglobin	14.8 g/dL
White Blood Cell	14,000/mL
Platelet	480,000/mL
Erythrocyte Sedimentation Rate	49 mm/hr.
C-Reactive Protein	20.4 mg/dL
Total Bilirubin	0.8 mg/dL
Albumin	4.8 g/dL
Alkaline Phosphatase	54 U/L
Gamma-glutamyltransferase	23 U/L
Alanine Transferase	16 U/L
Aspartate Transferase	20 U/L
Blood Urea Nitrogen	10 mg/dL
Creatinine	0.9 mg/dL
Sodium	135 mEq/L
Potassium	4.1 mEq/L
Chloride	103 mEq/L

Considering the physical examination and laboratory findings, the initial diagnosis was bacterial meningitis. Before performing the lumbar puncture, the patient was referred to undergo a computed tomography scan of the brain to rule out any space-occupying lesion and the risk of herniation. The head computed tomography scan demonstrated left tonsillar edema associated with ipsilateral filling defect in the internal jugular vein with stranding with the regional fat pads (Figure 1). Further, the thrombosis was extending to the left transverse dural venous sinus (Figure 2). In order to provide further evaluation, magnetic resonance imaging of the brain was requested. However, the patient was non-cooperative and had claustrophobia. Hence, the scan was performed with a single sequence of T1-weighted images with contrast enhancement. The scan showed intracranial dissemination of the disease with evidence of abscess formation (Figure 3). In view of the history of improperly treated pharyngitis, the radiological diagnosis was consistent with Lemierre’s syndrome.

**Figure 1:** Head CT shows tonsillar edema with thrombophlebitis involving the right internal jugular vein (arrow). CT: computed tomography

**Figure 2:** Head CT shows thrombosis of the right transverse dural venous sinus (arrow). CT: computed tomography

**Figure 3:** T1-weighted MR image with a contrast-enhancement shows cerebral abscess (arrow). MR: magnetic resonance

Subsequently, the patient was admitted to the intensive care unit on broad-spectrum intravenous antibiotics with piperacillin-tazobactam and clindamycin. The blood culture was positive for fusobacterium necrophorum. The antibiotic therapy was not changed since the organism was sensitive to the antibiotics started already. Anticoagulation with enoxaparin was given. The patient was kept on antibiotic therapy for a total of six weeks. He was discharged in a good condition with no residual deficits. After three months of follow-up, the patient had no complaints.

RETRACTED

## Discussion

We presented the case of a young adult with internal jugular thrombosis that developed after untreated pharyngeal infection, which is referred to as Lemierre’s syndrome. This syndrome is classically caused by Fusobacterium necrophorum, a gram-negative obligate anaerobic bacteria [5]. Lemierre’s syndrome is often referred to as a “forgotten disease” since the widespread antibiotic use in modern clinical practice led to a dramatic decrease in its incidence. As in the present case, Lemierre’s syndrome usually affects children and young adults with no previous medical conditions [6]. The estimated incidence of Lemierre’s syndrome currently is about three per 1,000,000 individuals every year [7].

The most frequent presenting symptom is a sore throat. In the present case, the sore throat preceded the neurological symptoms by two weeks. However, the average duration of the interval between the onset of fever and other symptoms is four days [5]. Further, fever is present in more than 90% of patients with Lemierre’s syndrome. Approximately 50% of patients have neck tenderness or mass [7]. In the present case, the patient had neck stiffness resulting from the meningeal irritation resulting from the intracranial dissemination of the disease. Septic embolism is common in Lemierre’s syndrome, including multifocal pneumonia, brain abscess, and septic arthritis. Pulmonary involvement is the most frequent and is noted in more than 80% of patients [6]. In our case, the initial chest x-ray showed no evidence of infiltrates to suggest pneumonia.

The most important clue to make the diagnosis of Lemierre’s syndrome is the finding of thrombophlebitis of the internal jugular vein [7]. A contrast-enhanced computed tomography scan is the best imaging investigation to evaluate for jugular vein thrombosis [5]. Magnetic resonance imaging is the investigation of choice to assess for suspected intracranial involvement. Furthermore, the growth of Fusobacterium necrophorum is another clue for the diagnosis. However, the identification of the organism may take up to seven days [6].

RETRACTED

Lemierre’s syndrome may have a mortality rate of more than 90% if left untreated [6]. However, even with the aggressive use of antibiotic therapy, it may have a mortality rate of up to 20% [5]. Disseminated intravascular thrombosis is a serious complication with associated poor outcomes [7]. In the present case, the coagulation profile of the patient was normal. However, the computed tomography scan indicated extension of the internal jugular vein thrombosis superiorly to involve the transverse dural venous sinus.

## Conclusions

Lemierre’s syndrome is a serious infection that develops after a pharyngeal infection. Considering the high mortality rate of untreated Lemierre’s syndrome, physicians should keep a high index of suspicion for this condition when they encounter a patient with upper respiratory tract infection with clinical or radiological findings consistent with internal jugular thrombophlebitis. The diagnosis is typically confirmed by imaging and the growth of Fusobacterium necrophorum in the bacterial culture. Aggressive parenteral antibiotics and systemic anticoagulation are the cornerstones of treatment.
